The article "Macrophages Mediate a Switch between Canonical and Non-Canonical Wnt Pathways in Canine Mammary Tumors" was retracted in 2019. Reasons: duplicated images; concerns about the data; concerns about the images.

# Macrophages Mediate a Switch between Canonical and Non-Canonical Wnt Pathways in Canine Mammary Tumors

**DOI:** 10.1371/journal.pone.0083995

**Published:** 2014-01-03

**Authors:** Magdalena Król, Joanna Mucha, Kinga Majchrzak, Agata Homa, Małgorzata Bulkowska, Alicja Majewska, Małgorzata Gajewska, Marta Pietrzak, Mikołaj Perszko, Karolina Romanowska, Karol Pawłowski, Elisabetta Manuali, Eva Hellmen, Tomasz Motyl

**Affiliations:** 1 Department of Physiological Sciences, Faculty of Veterinary Medicine, Warsaw University of Life Sciences, Warsaw, Poland; 2 Department of Animal Environment Biology, Faculty of Animal Sciences, Warsaw University of Life Sciences, Warsaw, Poland; 3 Department of Large Animal Diseases with Clinic, Faculty of Veterinary Medicine, Warsaw University of Life Sciences, Warsaw, Poland; 4 Area Diagnostica Integrata Istologia e Microscopia Elettronica Istituto Zooprofilattico Sperimentale dell'Umbria e delle Marche, Perugia, Italy; 5 Department of Anatomy, Physiology and Biochemistry, Swedish University of Agricultural Sciences, Uppsala, Sweden; Faculdade de Medicina, Universidade de São Paulo, Brazil

## Abstract

**Objective:**

According to the current hypothesis, tumor-associated macrophages (TAMs) are “corrupted” by cancer cells and subsequently facilitate, rather than inhibit, tumor metastasis. Because the molecular mechanisms of cancer cell–TAM interactions are complicated and controversial we aimed to better define this phenomenon.

**Methods and Results:**

Using microRNA microarrays, Real-time qPCR and Western blot we showed that co-culture of canine mammary tumor cells with TAMs or treatment with macrophage-conditioned medium inhibited the canonical Wnt pathway and activated the non-canonical Wnt pathway in tumor cells. We also showed that co-culture of TAMs with tumor cells increased expression of canonical Wnt inhibitors in TAMs. Subsequently, we demonstrated macrophage-induced invasive growth patterns and epithelial–mesenchymal transition of tumor cells. Validation of these results in canine mammary carcinoma tissues (n = 50) and xenograft tumors indicated the activation of non-canonical and canonical Wnt pathways in metastatic tumors and non-metastatic malignancies, respectively. Activation of non-canonical Wnt pathway correlated with number of TAMs.

**Conclusions:**

We demonstrated that TAMs mediate a “switch” between canonical and non-canonical Wnt signaling pathways in canine mammary tumors, leading to increased tumor invasion and metastasis.

Interestingly, similar changes in neoplastic cells were observed in the presence of macrophage-conditioned medium or live macrophages. These observations indicate that rather than being “corrupted” by cancer cells, TAMs constitutively secrete canonical Wnt inhibitors that decrease tumor proliferation and development, but as a side effect, they induce the non-canonical Wnt pathway, which leads to tumor metastasis.

These data challenge the conventional understanding of TAM–cancer cell interactions.

## Introduction

Interactions between various cell types within tumor microenvironments influence development, progression, and metastasis. Tumor-associated macrophages (TAMs), which reside in the tumor mass, play central roles in this intratumoral dialog [1], [2]. Indeed, the incidence of mammary tumors was much lower in macrophage-depleted mice than in normal mice, and metastasis was almost completely inhibited [3]. In patients with breast cancer, a positive correlation has been found between the density of TAMs and poor prognosis [3]–[5], and many *in vitro* and *in vivo* studies indicate that macrophages facilitate cancer metastasis [6]–[8]. Although several mechanisms have been proposed, most relate to the secretion by macrophages of various enzymes and metalloproteinases that facilitate matrix remodeling and thus influence the tumor microenvironment [9].

A prevalent hypothesis suggests that macrophages are corrupted by cancer cells and subsequently contribute to tumor progression instead of tumor inhibition [7], [10]. This mechanism comprises a paracrine signaling loop between tumor cells and TAMs that involves various chemokines and cytokines [9]. These factors secreted by cancer cells contribute to down-regulation of both expression of major histocompatibility complex class II and macrophage ability to present antigen. They also reduce TAM's antimicrobial and antitumoral activity and increase their production of pro-angiogenic factors, such as vascular endothelial growth factor [11]. In addition, “corrupted” TAMs secrete various growth factors that facilitate the spread of cancer cells into blood vessels, lymph nodes, and distal organs [11].

Interestingly, Pukrop et al. [12] suggested that TAMs influence the tumor microenvironment by modulating Wnt signaling. They showed that TAMs secrete Wnt-5a, which induces MMP-7 expression in cancer cells and facilitates successful invasion. More recently, Oljavo et al. [9] examined Wnt signaling in the cancer microenvironment and showed that TAMs secrete Wnt-7b, which enhances vasculogenesis. Moreover, our previous microarray analyses showed increased *Wnt-5b, Wnt-7a*, and *Wnt-7b* expression in macrophages during co-culture with cancer cells [8].

The Wnt signaling pathway is critical for development, cell motility, invasion, angiogenesis, and tissue repair. However, its inappropriate activation is responsible for the development of diseases such as cancer [13]. The canonical Wnt pathway involves β-catenin, which acts as a transcription factor for increased cell proliferation and survival after translocation from cellular membranes to the nucleus [13]. Non-canonical Wnt pathways, Ca^2+^-dependent and planar cell polarity (PCP) signaling, activate PKC and JNK/small Rho-GTPases, respectively. These pathways regulate cytoskeletal architecture, increase cell invasion and migration, and decrease proliferation by inhibiting the canonical Wnt pathway [13].

As stated above, the molecular mechanisms of cancer cell–TAM interactions are complicated and controversial. Thus, to investigate the interactions between macrophages and cancer cells, we performed microarray analyses of miRNA expression in co-cultures of canine mammary tumor cells and macrophages.

The present observations provide new insights into the interactions between neoplastic cells and macrophages in the tumor microenvironment.

## Materials and Methods

### Cell lines, culture and co-culture conditions, and cell sorting

#### Canine mammary tumor cell lines

Cell lines were described in our previous studies [8], [14]. In brief, two canine mammary carcinoma cell lines (CMT-W1, CMT-W2) were kindly donated by Prof. Dr. Maciej Ugorski (Wrocław University of Environmental and Life Sciences, Poland), an anaplastic cancer cell line (P114) was kindly donated by Dr. Gerard Rutteman (Utrecht University, The Netherlands), a simple carcinoma cell line (CMT-U27), and a spindle cell mammary tumor cell line of epithelial origin (CMT-U309) were kindly donated by Prof. Dr. Eva Hellmen (Swedish University of Agricultural Sciences, Sweden). Cells were cultured in RPMI 1640 medium supplemented with 10% (v/v) heat-inactivated fetal bovine serum, penicillin-streptomycin (50 IU/mL), and fungizone (2.5 mg/mL; Sigma Aldrich, USA) in an atmosphere of 5% CO_2_ and 95% humidified air at 37°C [8], [14].

#### Macrophages

Macrophages were cultured as described previously [8]. In brief, anti-coagulated whole blood was collected from healthy dogs for routine diagnostic purposes or for deposition in a blood bank. The owners of the dogs gave permission for their animals to be used in this study. Samples were immediately subjected to mononuclear cell separation using Accuspin System-Histopaque 1077 (Sigma Aldrich), according to the manufacturer's protocol. Isolated mononuclear blood cells were incubated for 1 h at room temperature with mouse monoclonal anti-CD64 FITC-conjugated (BD Biosciences, USA) antibodies, according to the manufacturer's instructions (20 µL/10^6^ cells). Monocytes were initially identified and gated on the basis of morphological criteria (SSC vs FSC cytogram) using FACSAria II (BD Biosciences). Subsequently, CD64-positive cells were gated, sorted, and co-cultured with cancer cells or as monocultures supplemented with 25 µg/mL CSF-1 [13].

#### Co-culture and sorting

In this model, neoplastic cell lines (CMT-W1, CMT-W2, CMT-U27, CMT-U309, and P114) were grown in separate flasks, and sorted monocytes were then layered onto the cancer cell monolayers at a ratio of 1∶5, as described previously [8]. In brief, the Orange CellTracker fluorescent dye CMTMR (Invitrogen, USA) was used at 5 µM to stain neoplastic cells prior to the addition of sorted monocytes. Co-cultures were maintained for 72 h, harvested by trypsynization, stained with anti-CD-64 antibodies (BD Biosciences), and sorted into two tubes of CD-64-positive/CMTMR-negative macrophages and CMTMR-positive/CD-64-negative neoplastic cells using FACSAria II. In agreement with a previous study [8], no significant differences in red dye optical density in tumor cells were observed between confocal microscopy analyses performed immediately and 72 h after staining, indicating no leakage of dye from neoplastic cells. Indeed, comparisons of red dye fluorescence with observations made using Nomarski Interference Contrast (NIC) showed that the cells maintained their staining pattern for at least 72 h. FACS sorting isolated a 97–99% pure population on the post-sort, as assessed using BD FACS Diva version 5.0 software and confirmed using fluorescence microscopy [8]. Thus, contamination of neoplastic cells with macrophages was improbable but cannot be completely ruled out. Previous studies show successful experiments with cells sorted from direct co-culture of neoplastic cells and macrophages [8], [9]. However, to confirm that the effects of macrophages on tumor cells were not due to macrophage contamination of sorted cancer cells, we treated neoplastic cells with macrophage-conditioned medium.

#### Cancer cell culture in macrophage-conditioned medium

Macrophage-conditioned medium was collected, centrifuged, filtered, and stored in aliquots at −20°C. These aliquots were then added to cancer cell medium at 20%; equivalent to the ratio of macrophages and tumor cells (1∶5) in co-cultures.

### miRNA microarray analysis

Total-RNA (t-RNA) was isolated from samples using a Micro RNA kit (A&A Biotechnology, Poland), according to the manufacturer's protocol. The quantity of t-RNA was measured using a NanoDrop instrument (NanoDrop Technologies, USA), and final RNA quality and integrity were assessed using a BioAnalyzer (Agilent, USA). Only high-quality samples (RIN>8) were used in further analyses.

A microRNA Labeling & Hybridization Kit (Agilent) was used to amplify and label mature miRNAs for microarray experiments. The canine miRNA microarray containing 323 miRNA sequences was custom designed using an eArray Agilent online service, and all sequences from miRBase 17.0 were included. This microarray platform has been deposited in NCBI's Gene Expression Omnibus and is accessible via the GEO Series accession number GPL16580.

miRNA expression in tumor cells sorted from co-culture with macrophages was compared with that in monocultures. miRNA expression in macrophages sorted from co-culture with tumor cells was compared with that in monocultured macrophages. Each sample was examined eight times. Acquisition and analysis of hybridization intensities were performed using a DNA microarray scanner (Agilent), and data were extracted using Agilent's Feature Extraction software with normalization and robust statistical analyses.

#### Biostatistical analysis

Statistical analyses were performed using Future Extraction and Gene Spring software (Agilent). Unpaired t-tests with a Benjamin–Hochberg false discovery rate (FDR) of <5% correction were applied, with a p value cut-off of <0.01. Only miRNAs that were significantly regulated by co-culture conditions in all neoplastic and macrophage samples were analyzed. Significantly regulated miRNAs were selected from eight technical and five biological repetitions (five cell lines). Areas of these analyses have been deposited in NCBI's Gene Expression Omnibus and are accessible using the GEO Series accession number GSE43968.

Genes targeted by miRNA were analyzed using miRBase, and corresponding signaling pathways were identified using PANTHER pathway analysis software [15].

### Real-time RT-PCR

Real-time RT-PCR analyses were used to validate microarray data. Total RNA was reverse transcribed using Universal cDNA synthesis kit II (Exiqon, USA), and cDNA was synthesized. Quantitative RT-PCR was performed using a fluorogenic SYBR Green Master Mix kit (Exiqon) and a Mx3005P QPCR System (Agilent). Commercially available microRNA LNA PCR primer sets (Exiqon) were used to amplify miR-130a and miR-182, and data were expressed relative to spike-in controls. Data were analyzed using the comparative Ct method [16]. The experiment was repeated five times.

Sequences of key genes were obtained from the NCBI database. Primers were designed using Primer3 software (free online access) and were checked using Oligo Calculator (free online access) and Primer-Blast (NCBI database). Primer sequences are listed in Table 1. The housekeeping genes *Hprt* and *Rps19* were used as internal controls [17], [18]. Quantitative RT-PCR was performed using a fluorogenic Lightcycler Fast Strand DNA SYBR Green kit (Roche) and a Light Cycler (Roche). Data were analyzed using the comparative Ct method [16]. The experiment was repeated five times.

**Table 1:** Primer's sequences used in this study and their annealing optimal temperature and time.

Gene name	Left Primer	Right Primer	Annealing temp	Annealing time
***Axin 2***	CCCACCTTGAATGAGGAAGA	GTCTCCGTGGACCTCACATT	60	4
***Ccn D1***	ACGTGAACATTTGAGGGTGC	AGACGGAAGGGAGAAAGAGC	61	6
***Cd 163***	ATGTCCAGTGTCCAAAAGGA	CATGTGATCCAGGTCTCCTC	61	6
***Ctnn B1***	GCTGTTCGCCTTCACTATGG	TCCACCCATAGATGTACGGC	61	8
***Dkk1***	CTTCCATCGAGGAGAGATCG	TTTCGAAGACAGGGTGGTTC	60	4
***Lrp6***	CCCGGAGAAGGGGTATATGT	AAAGCTTGCCCAATCTGCTA	60	6
***Mmp9***	CGACTACGACCAGGACAAAC	AAGCCCCACTTCTTGTCTCT	61	8
***Tbl1X***	TGATCTCGGCCTCCACATAC	TCCCGCATCATACAGACCTC	60	9
***Tbl1xR1***	ATTGCACTAACCTCCCTGCT	CCCGTGCTATCATTTGCGAA	60	10
***TGFB1R1***	GATGGGCTCTGCTTTGTCTC	CCTGGTTGCAGCAATAGGTT	61	6
***Wnt-2***	GCATCCTTTCCCTTCCTTTC	TCAGCTGGAGTTGTGTTTGC	60	8
***Wnt-2b***	CCTCAACTCTGGGCTGCTAC	TCAGGGAGCCATTCAATTTC	60	6
***Wnt-3***	TGGACCACATGCACCTTAAA	CTTGAGGAAGTCGCCGATAG	60	4
***Wnt-5a***	TGCCACTTGTATCAGGACCA	GCTGCCTATCTGCATGACC	61	10
***Wnt-5b***	CCCTGTACAGAGACCCGAGA	CACTCCTTGATGCCCGTCTT	60	6
***Wnt-7a***	CAACCTGAGTGACTGTGGCT	CCGCCTCGTTATTGTGCAAG	61	6
***Wnt-7b***	GCGGAGGGCTGTGTATAAGA	GTCCCCTACTTTGCGGAACT	61	10
***Rps19***	CCTTCCTCAAAAAGTCTGGG	GTTCTCATCGTAGGGAGCAAG	61	10
***Hprt***	AGCTTGCTGGTGAAAAGGAC	TTATAGTCAAGGGCATATCC	59	6

The mRNA sequences of key genes were obtained from NCBI database. Primers were designed using PRIMER3 software (free on-line access) and checked using Oligo Calculator (free on-line access) and Primer-Blast (NCBI database).

PCR products were electrophoresed through ethidium bromide-stained 2% agarose gels (Sigma Aldrich) for 60 min at 90 mV in Tris-borate-EDTA buffer. The gels were then visualized under UV light [19].

### Western blotting

Protein expression was assessed using western blotting. Control tumor cells, tumor cells grown in macrophage-conditioned medium, tumor cells sorted from co-culture with macrophages, and macrophages from monocultures and sorted from co-culture with tumor cells were analyzed.

The cells were pelleted by centrifugation at 400 *g* for 5 min at 4°C. Nuclear and cytoplasmic protein extracts from cultured cells were isolated by lysis using the CelLytic NuCLEAR reagent (Sigma Aldrich), according to the manufacturer's instructions. Total protein concentrations in lysates were determined using a Bio-Rad protein assay (Bio-Rad Laboratories Inc., USA). Proteins (50 µg) were resolved using SDS-PAGE and transferred onto PVDF membranes (Sigma Aldrich). The membranes were then blocked with 5% non-fat dry milk in TBS buffer containing 0.5% Tween 20. The membranes were then incubated overnight with the primary anti-canine antibodies anti-Wnt-2, anti-Wnt-5a, anti-Dkk-1, anti-p-JNK1/3, anti-JNK1/3, anti-p-PKC α/β II, anti-PCK (Bioss, USA), anti-Lamin a/c, anti-ROR-2 (Pierce, USA), anti-p-Akt and anti-Akt (SantaCruz Biotechnology Inc., USA), anti-β-catenin (GeneTex, USA), anti-calmodulin, and anti-β-actin (Milipore, USA) at 4°C. Subsequently, the membranes were washed three times in TBS containing 0.5% Tween 20 and incubated for 1 h at room temperature with secondary antibodies conjugated with the appropriate infrared (IR) fluorophore IRDye® 800 CW or IRDye® 680 RD at a dilution of 1∶5000. An Odyssey Infrared Imaging System (LI-COR Biosciences, USA) was then used to analyze protein expression. Scan resolution and intensity of the instrument were set at 169 µm and 4, respectively. Quantification of the integrated optical density (IOD) was performed using the analysis software provided with the Odyssey scanner (LI-COR Biosciences). To remove antibodies, the membranes were incubated for 15 min at room temperature in Restore Western Blot Stripping Buffer (Thermo Scientific, USA). This experiment was repeated seven times.

### Cell viability assay (MTT assay)

Cell viability (metabolic activity of viable cells) was quantified using MTT assays. In brief, the cells were seeded onto 96-well plates (Nunc Inc., Denmark) at 1×10^4^ cells/well. On the following day, the medium was replaced with medium containing 20% macrophage-conditioned medium or with macrophages at a ratio of 1∶5 tumor cells. The cultures were incubated for 72 h, and the cells were incubated with 0.5 mg/mL of the tetrazolium salt MTT diluted in phenol red-free RPMI 1640 medium (Sigma Aldrich) for 4 h at 37°C. To complete solubilization of formazan crystals, 100 µL of dimethyl sulfoxide (Sigma Aldrich) was added to each well. Cell viability was quantified by measuring photometric absorbance at 570 nm using a multiwell plate reader (Infinite 200 PRO Tecan™, TECAN, Switzerland). All samples were examined nine times.

### Immunohistochemical (IHC) examination of canine mammary neoplastic cell lines, cancer tissues, and xenograft tumors

Cell lines and macrophages were cultured on Lab-Tek 4-chamber culture slides (Nunc Inc., USA) for 24 h and were subjected to IHC analysis after ethanol (70%) fixation for 10 min.

Canine mammary tumor tissue sections were derived from the archives of the Department of Pathology and Veterinary Diagnostics, Faculty of Veterinary Medicine, Warsaw University of Life Sciences (Poland) and Area Diagnostica Integrata Istologia e Microscopia Elettronica, Istituto Zooprofilattico Sperimentale dell'Umbria e delle Marche (Italy). Samples were surgically collected during mastectomy from 50 female dogs of various breeds. Tissue samples were fixed in 8% neutral buffered formalin and routinely embedded in paraffin. Tumor samples included diagnosed malignant non-metastatic (n = 25) and malignant metastatic (n = 25) carcinomas. Metastatic tumors were surgically removed with their metastatic sites. The presence of neoplastic cells in metastatic site was histologically confirmed using hematoxylin and eosin (HE)-stained slides. The tumors were diagnosed according to the World Health Organization Histological Classification and Mammary Tumors of the Dog and Cat classification [20].

The xenograft tumors grew due to CMT-U27 cells inoculation in 8-week-old male athymic nude mice (Balb/c nu/nu) [20] were analyzed. The cells were suspended in PBS at 4×10^6^ cells/0.1 mL and inoculated subcutaneously into the necks of mice. Upon metastasis into lymph nodes [21], tumors were surgically removed and fixed in paraffin blocks. Male mice were selected for this study to avoid hormonal influence [22].

Sections of 4 µm were taken from paraffin tumor tissue blocks and were incubated overnight at 37°C. After dewaxing in xylene and rehydration in ethanol, antigens were retrieved by placing slides in 0.02 M citrate buffer (pH 6.0) and boiling in a decloaking chamber.

Samples were incubated in a peroxidase blocking reagent (Dako, Denmark) for 10 min at room temperature prior to 30 min incubation in 5% bovine serum albumin (Sigma Aldrich, Germany). Then, the primary anti-canine antibodies anti-β-catenin (1∶100 dilution; GeneTex), anti-Wnt-2, anti-Wnt-5a, anti-Dkk-1 (1∶200 dilution; Bioss), anti-ROR-2 (1∶200 dilution; Pierce) were diluted in 1% bovine serum and were applied to cells overnight at 4°C. Cell lines were incubated with 1∶100 dilutions of anti-cytokeratin (clone AE1/AE3), anti-vimentin, or anti-MAC387 (Dako) antibodies for 1 h at room temperature. Subsequently, an Envision kit comprising labeled polymers of secondary anti-rabbit/mouse antibodies conjugated with the HRP enzyme complex (Dako) was used. The 3,3′-diaminobenzidine (Dako) substrate was used to develop colored products. Finally, nuclei were counterstained with hematoxylin. Each IHC experiment was controlled by omitting primary antibodies on representative paraffin slides.

Three consecutive tissue sections and four slides of each cell line were analyzed. Pictures of each slide were taken (10–20 depending on the sample size) using an Olympus BX60 microscope. Colorimetric intensities of IHC-stained antigen spots (brown precipitate reflecting antigen expression) were counted using a computer-assisted image analyzer (Olympus Microimage™ Image Analysis version 4.0 software for Windows, USA). The intensities of color related to each antigen spot were expressed as mean pixel IOD. Β-catenin localization was observed as nuclear, cytoplasmic, or membranous.

### Culture on Matrigel matrix

Culture plates (35 mm; Corning Inc.) were coated with 100 µL of growth factor-reduced Matrigel (BD Biosciences) and were left to solidify for 30 min at 37°C. The cells were then plated at a concentration of 10^4^ cells/mL and cultured in normal or macrophage-conditioned medium. Cell growth on Matrigels was observed everyday using a phase contrast microscope.

### Confocal microscopy

Control canine mammary tumor cells, tumor cells cultured in macrophage-conditioned medium, and co-cultured with macrophages were seeded on Lab-Tek slides (previously coated with Matrigel) for 72 h. The cells were then washed two times in warm PBS and were fixed in 3.7% paraformaldehyde for 20 min at room temperature. Subsequently, the cells were permeabilized with 0.5% Triton X-100 diluted in PBS for 10 min at room temperature, washed three times in PBS, and incubated with rabbit anti-phospho-fascin (FSCN1, Ser39) antibodies diluted 1∶100 in PBS (Bioss). After overnight incubation with primary antibodies at 4°C, the cells were washed three times in PBS, incubated with secondary Alexa Fluor 568 goat anti-rabbit antibodies (diluted 1∶500 in PBS; Santa Cruz Biotechnology Inc.), and stained for F-actin using FITC–X phalloidin (diluted 1∶100 in PBS; Invitrogen) for 1 h in the dark at room temperature. Coverslips were then mounted on microscope slides using mounting medium (Sigma Aldrich). Cell imaging was performed using a confocal laser scanning microscope FV-500 system (Olympus Optical Co., Germany) with an 488-nm argon laser and 505- to 525-nm filter for FITC staining and with a 543-nm He-Ne laser and a 610-nm filter for Alexa Fluor 568 staining. Images were gathered separately for each fluorescence channel, and the cells were examined using the Fluoview program (Olympus Optical Co.).

### Statistical analysis

Statistical analyses were performed using Prism version 5.00 software (GraphPad Software, USA). Two-way analysis of variance (ANOVA), ANOVA with Tukey's honestly significant difference post-hoc test, t-test, and Spearman's correlation were applied, and differences were considered significant when p<0.05 or highly significant when p<0.01 or p<0.001.

## Results and Discussion

### Co-culture of tumor cells and macrophages caused significant changes in miRNA expression in both cell types

Molecular interactions between various components of the tumor microenvironment remain unclear. Thus, to elucidate mechanisms by which macrophages and cancer cells influence each other, we initially performed microarray analysis of miRNA expression in co-cultured canine mammary tumor cells and macrophages. Microarray experiments revealed 143 tumor cell miRNAs that were significantly regulated by co-culture with macrophages and 264 miRNAs that were significantly regulated in co-cultured macrophages (p<0.01, fold change >1.2) (Table 2). We randomly selected two miRNAs and using real-time RT-PCR, we validated these microarray results and confirmed that co-culture resulted in a 4-fold increase (p<0.01) and a 10-fold decrease (p<0.001) in miR-182 expression in macrophages and tumor cells, respectively. We also observed a 23-fold increase (p<0.001) and a 439.5-fold decrease (p<0.001) in miR-130a expression in co-cultured macrophages and tumor cells, respectively (Figure S1). Using miRBase we found target genes for the miRNAs listed in Table S1. Then, we analyzed functions of these genes using PANTHER database. We revealed that Wnt signaling predominated in both co-cultured cell types (p<0.01). Analysis of the list of miRNA-targeted Wnt genes indicated that co-culture conditions mainly induced expression of canonical Wnt inhibitors and non-canonical Wnt ligands (Table 2 and Table S2). In cancerneoplastic cells co-cultured with macrophages we showed up-regulation of miRNAs targeting *Axin 1*, *CcnD1, Ctnnb1, Tbl1xr1*, *Dkk-1*, *Wnt-2*, *Wnt-7b*, *Wnt-8b* and *Wnt-10a* genes and down-regulation of *Axin 2*, *Lrp 6*, *Wnt-3*, *Wnt-4*. These changes might indicate a “switch” from canonical Wnt pathway to non-canonical Wnt pathway. In macrophages co-cultured with tumor cells we showed down-regulation of miRNAs targeting: *Axin 1*, *Axin 2*, *Lrp6*, *Wnt-2b*, *Wnt-4*, *Wnt-5a*, *Wnt-7b*, *Wnt-8b*, *Wnt-10a* and *Wnt-10b*. Taken together, we showed tumor cell-mediated increase in expression of canonical Wnt inhibitors and non-canonical Wnt ligands in macrophages. Next, we aimed to confirm these observations.

**Table 2:** The list of Wnt-targeting miRNAs regulated in canine mammary cancer cell lines and macrophages grown as a co-culture. Table is based on microarray data and miRBase.

Wnt target gene	miRNA regulated in cancer cells grown with macrophages		miRNA regulated in macrophages grown with cancer cells	
	up	down	up	down
***Axin 1***	miR-124, miR-137, miR-212, miR-377		miR-141	miR-128
***Axin 2***	miR-15a	miR-183		miR-103, miR-107, miR-221, miR-222, miR-301a, miR-340
***Ccn D1***	miR-495			miR-219
***c-JUN***	miR-144	miR-24		miR-101, miR-30e
***Ctnn A1***	miR-181b	miR-181d		miR-30b
***Ctnn B1***	miR-150, miR-214, miR-219, miR-382, miR-496, miR-543	miR-181d		miR-320
***Dkk 1***	miR-219			miR-219
***Lrp 5***		miR-346		
***Lrp 6***	miR-202, miR-377	let-7a, let-7b, miR-183		let-7b, let-7c, miR-194, miR-27a, miR-27b, miR-497
***NLK***		miR-183		miR-140, miR-33a
***Tbl1xR1***	miR-133a, miR-133b, miR-181d	miR-135b	miR-141, miR-200c	miR-148a, miR-148b, miR-181a, miR-186, miR-505
***Wnt-2***	miR-139, miR-217		miR-130a	
***Wnt-2b***	miR-217	miR-24		miR-24, miR-30c
***Wnt-3***	miR-136	miR-135b, miR-24, miR-33b		miR-19b, miR-21, miR-210, miR-324, miR-542
***Wnt-4***	miR-133a, miR-181d, miR-376c	miR-130a, miR-151, miR-24	miR-130a, miR-365	miR-151, miR-181d, miR-195, miR-24, miR-26a, miR-30e, miR-362, miR-374a, miR-374b, miR-425, miR-497, miR-551b
***Wnt-5a***	miR-181b, miR-212, miR-31	miR-23a, miR-24		miR-126, miR-140, miR-146b, miR-181a, miR-185, miR-31, miR-324
***Wnt-7b***	miR-153, miR-153, miR-181b, miR-31	miR-183		miR-146a, miR-181a, miR-22, miR-221, miR-26a, miR-27b, miR-301a, miR-30c, miR-31, miR-32, miR-324, miR-361
***Wnt-8b***	miR-127, miR-369			miR-186, miR-195, miR-27b, miR-30c, miR-33a
***Wnt-10a***	miR-133b, miR-145			let-7c
***Wnt-10b***				miR-185, miR-210

The area of the analyses covered in this publication has been deposited in NCBI's Gene Expression Omnibus and is accessible via GEO Series accession number GSE43968.

Although this study indicated epigenetic regulation of neoplastic cells by macrophages and *vice versa*, these results also offer a method for screening pathways that are significantly regulated in co-cultures of tumor cells and TAMs.

### Macrophages induced a switch between canonical and non-canonical Wnt signaling

We performed real-time RT-PCR and western blot analyses of selected miRNA targets to confirm the inhibition of the canonical Wnt pathway and the activation of the non-canonical Wnt pathway in neoplastic cells co-cultured with TAMs (Figure 1, Figure 2, Figure S2 and Table 3). Because the strongest effects were observed in CMT-U27, CMT-U309, and P114 cell lines, further experiments were performed using these three cell lines alone. We confirmed that co-cultured macrophages differentiated into TAMs (M2 macrophages), as indicated by the increased expression of the TAM-specific markers *Cd163* and *Mmp9* (Figure 1A) [23]. Macrophages can differentiate toward M1 (classically activated by LPS) or M2 (TAMs, alternatively activated often by tumor hypoxia or selected interleukins) phenotypes [24]. The present experiments show that culture of macrophages in CSF-1 (control macrophages) maintained their proliferation but did not induce polarization (Figure 1A).

**Figure 1:** Expression of selected Wnt genes in co-cultured canine mammary tumor cells and macrophages. Real-time RT-PCR analysis of Wnt genes in co-cultured and monocultured canine mammary neoplastic cells and macrophages. (A) Representative agarose gel electrophoresis of *Cd163* and *Mmp9* PCR products following real-time SYBR Green amplification in macrophages cultured alone and in co-culture with neoplastic cells. (B) Representative agarose gel electrophoresis of PCR products following real-time SYBR Green amplification (CA, cancer cells grown as monoculture; CA+MQ, co-cultured cancer cells; MQ, mono-cultured macrophages; and MQ+CA, macrophages co-cultured with cancer cells). (C) Fold changes in examined genes in co-cultured macrophages compared with control macrophages. (D) Western blots of cytoplasmic and membrane Wnt proteins from Macrophages grown as monocultures or sorted from co-culture with canine mammary neoplastic cells. The level of examined proteins (E, F, G) was expressed as IOD (Integrated Optical Density) in arbitrary units with the value obtained using the Odyssey Infrared Imaging System (LI-COR Inc., USA). The results are expressed as the mean ±SD. The ANOVA + Tukey post-hoc test were applied (Graph Pad v. 5.0), the values differed significantly (p<0.05) were marked as *, whereas values differed highly significant (p<0.01 or p<0.001) were marked as ** or ***, respectively.

**Figure 2:** Expression of Wnt proteins in co-cultured canine mammary tumor cells and macrophages. Fold changes of Wnt genes in CMT-U27, CMT-U309, and P114 canine mammary neoplastic cells cultured in macrophage-conditioned medium or co-cultured with macrophages compared with control cells (A). Analysis of variance and Tukey's test were applied (GraphPad Prism 5.0, USA); the Differences were considered significant when *p<0.05 and highly significant when **p<0.001. Western blots of cytoplasmic and membrane or nuclear (**B**) Wnt proteins from CMT-U27, CMT-U309, and P114 canine mammary neoplastic cells grown in control medium, macrophage-conditioned medium, or in co-culture with macrophages. (**C**) Neoplastic cell survival (MTT assays) in control media, macrophage-conditioned medium (CM) and in co-culture with macrophages (MQ).

**Table 3:** The β-catenin staining pattern, number of tumor associated macrophages (TAMs) and expression (IOD, Integrated Optical Density) of Wnt-2, Wnt-5a, Dkk-1 and ROR-2 in canine mammary metastatic and non-metastatic tumors.

B-catenin staining pattern	metastatic tumors	non-metastatic tumors
Nucear		N = 5
nucelear+cytoplasmic		N = 13
nucear+cytoplasmic+membranous		N = 5
cytoplasmic+membranous	N = 2	N = 2
cytoplasmic	N = 23	
Number of TAMs	115 (±10)	80 (±8)
IOD of Wnt-2	550,000 (±8,663)	181,750 (±120,550)
IOD of Wnt-5a	511,300 (±201,236)	109,284 (±5,352)
IOD of Dkk-1	174,456 (±50,231)	85,053 (±31,837)
IOD of ROR-2	516,667 (±125,831)	233,333 (±76,376)

In TAMs, we showed significant upregulation of genes encoding the highly potent canonical Wnt inhibitor *Dkk-1* [25], non-canonical activators *Wnt-5a* and *Wnt-2a*, and non-canonical ligands *Wnt-5b*, *Wnt-3*, *Wnt-7a*, and *Wnt-7b* (Figure 1B and C) [9]. Moreover, the expression of the canonical Wnt receptor *Lrp6* was significantly decreased in TAMs compared with control macrophages, and the expression of the canonical Wnt inhibiting receptor *Tblx1r* was significantly increased [13]. Wnt-2, Wnt-5a, and Dkk-1 proteins were expressed at very low levels under control conditions, and their expression was significantly increased in co-cultured TAMs (Figure 1D-G). Control macrophages constitutively secreted non-canonical Wnt activators, and co-culture with neoplastic cells induced further secretion of these proteins. Thus, we suggested that cancer cells may not corrupt macrophages because they secrete the same key Wnt proteins when cultured alone or with neoplastic cells.

In contrast, the presence of macrophages in the tumor cell microenvironment caused significant changes in the expression of Wnt genes (Figure 1B, Figure 2A). Upon co-culture with macrophages, we observed *Axin2* (which facilitates β-catenin degradation), *Dkk-1*, *Wnt-2*, *Wnt-2b*, *Wnt-3*, *Wnt-5a*, and *Wnt-7a* upregulation and *Cyclin D1*, *β-catenin*, and *Lrp6* downregulation in tumor cells (Figure 1B; Figure 2A). Increased expression of Wnt-2, Wnt-5a, and Dkk-1 proteins was also confirmed in these cells (Figure 2B, Figure S2). Moreover, treatment of tumor cells with macrophage-conditioned medium caused similar changes in mRNA and protein expression of examined Wnt genes and proteins (Figure 2A, B, Figure S2). We observed that in neoplastic cells nuclear and cytoplasmic level of β-catenin decreased in the presence of macrophage-conditioned medium or TAMs (Figure 2B, Figure S1), further indicating the inhibition of canonical Wnt signaling [13].

To our knowledge, only one previous study described the changes in the expression of Wnt ligands in indirectly co-cultured macrophages and cancer cells [12]. The authors reported Wnt-5a mRNA upregulation in macrophages during co-culture with MCF7 breast cancer cells. However, no concomitant changes were observed in the expression of other Wnt genes [12]. Importantly, the Wnt genes examined by these investigators were significantly different from those examined in the present study. In our opinion differences between direct and indirect exposure to macrophages could not account for these discrepancies because the effects of co-culture with macrophages and macrophage-conditioned medium were comparable.

Our western blot analyses of downstream Wnt signaling confirmed the inhibition and activation of canonical and non-canonical Wnt pathways, respectively, in tumor cells exposed to TAMs or macrophage-conditioned medium. Indeed, we observed decreased AKT phosphorylation in these tumor cells (Figure 2B, Figure S2) confirming canonical Wnt pathway inhibition [26]).

We revealed Ca^2+^-dependent non-canonical Wnt signaling activation in tumor cells exposed to macrophage-conditioned medium or TAMs, as indicated by increased PKC A/B phosphorylation and increased calmodulin expression (Figure 2B, Figure S2). Based on the literature data increased PKC phosphorylation and calmodulin expression may be markers of Ca^2+^-dependent non-canonical Wnt signaling activation [13], [27].

We also observed the activation of the non-canonical PCP Wnt signaling pathway, with macrophage-conditioned medium and TAM-induced phosphorylation of JNK 1/3 and induction of the Wnt-5a receptor ROR-2 (Figure 2B, Figure S2). Based on the literature data increased phosphorylation of JNK 1/3 and increased expression of ROR-2 may be markers of PCP Wnt signaling pathway activation [28].

Given the similar, albeit less significant, effects of macrophage-conditioned medium and co-culture with TAMs, corruption of macrophages by cancer cells may not be necessary for their contribution to tumor progression. Indeed, this observation suggests the constitutive macrophage expression of canonical Wnt pathway inhibitors. Hence, whereas macrophage-derived canonical Wnt inhibitors may inhibit cancer cell proliferation, they may also facilitate metastasis by activating the non-canonical Wnt pathway. Accordingly, tumor cell proliferation was significantly decreased in the presence of macrophage-conditioned medium or TAMs (Figure 2C), with 20% inhibition of CMT-U27 cell proliferation (p<0.05) in the presence of macrophage-conditioned medium and 40% inhibition in the presence of live macrophages (p<0.001). In CMT-U309 cells, the addition of macrophage-conditioned medium and TAMs resulted in 22% and 32% decreases in cell proliferation (p<0.05), respectively. Strikingly, P114 cell proliferation was reduced by almost 50% in the presence of macrophage-conditioned medium (p<0.001) and by 62% in co-culture with macrophages (p<0.001). To proof this hypothesis we examined changes in cytoskeleton of tumor cells due to co-culture with macrophages or treatment with macrophage-conditioned medium.

### Cytoskeleton rearrangement

Analysis of changes in tumor growth patterns on Matrigel matrix showed that monocultured neoplastic cells formed unbranched colonies. In contrast, incubation with macrophage-conditioned medium (Figure 3) or TAMs [8] for 72 h led to the formation of branches and invasion of the Matrigel matrix.

**Figure 3:** Growth characteristic on the Matrigel matrix. Phase contrast micrographs of CMT-U27, CMT-U309, and P114 cells grown on the Matrigel matrix for 72 h under control conditions or in macrophage-conditioned medium. Control neoplastic cells formed colonies, whereas those treated with macrophage-conditioned medium invaded the Matrigel matrix and formed branches.

Using confocal microscopy, we studied cytoskeletal rearrangements in the context of F-actin and fascin-1 cross-linking and filopodia formation [29]–[31]. As illustrated in Figure 4A, fascin-1 was poorly co-localized with F-actin in control cells, and was centrally localized. After incubation of cancer cells in macrophage-conditioned medium for 72 h, the distribution of phosphorylated fascin-1 became more diffuse in the cytoplasm, but was observed in filopodia and at cell edges (Figure 4B). Activation of the Ca^2+^-dependent Wnt pathway leads to the phosphorylation of fascin-1 and formation of complexes with PKC [32] at cell edges. This is necessary for directional cell migration and metastasis [32]. This effect was increased after co-culture with macrophages for 72 h, and stress fiber formations were observed (Figure 4C), indicating the activation of the PCP Wnt signaling pathway.

**Figure 4:** Confocal and immunohistochemical analysis of canine mammary tumor cell lines grown in co-culture with macrophages. Confocal images show expression, distribution, and co-localization of actin and p-FSCN1 and formation of stress fibers in control (**A**), conditioned medium-treated (**B**), and co-cultured (**C**) CMT-U27 canine mammary cancer cells. Graph (**D**) and representative pictures (**E**) of cytokeratin and vimentin expression in control canine mammary cancer cells (CMT-U27) and after culture in macrophage-conditioned medium (MC-medium) or co-culture with macrophages. Monocultured neoplastic cells showed strong cytokeratin expression and weak vimentin expression. Cytokeratin expression was significantly weaker due to culture in macrophage-conditioned medium or co-culture with macrophages. On the other hand, vimentin expression was found to be significantly stronger due to neoplastic cell culture in macrophage-conditioned medium or co-cultured with macrophages. Cytokeratin (CK) and vimentin (VIM) expression was examined in control macrophages (**F**; graph and representative pictures). They showed no expression of cytokeratin whereas they showed vimentin expression at the same level as neoplastic cells grown in macrophage-conditioned medium (no significant difference). Images were generated using an Olympus BX60 microscope (200×); Cytokeratin and vimentin are indicated by brown precipitates.

### Macrophages drive epithelial–mesenchymal transition in cancer cells

Non-canonical Wnt signaling is responsible for the epithelial–mesenchymal transition (EMT) in *Drosophila melanogaster* [33], [34], which is crucial to cancer invasiveness and metastasis [34]. In the present study, control tumor cells showed significantly higher expression of the epithelial marker cytokeratin than neoplastic cells cultured in macrophage-conditioned medium or co-cultured with macrophages (Figure 4D, E). Tumor cells cultured in macrophage-conditioned medium or co-cultured with macrophages also had significantly increased expression of the mesenchymal marker vimentin compared with control cells. As a control, we examined level of cytokeratin and vimentin expression in macrophages. In control macrophages we showed no expression of cytokeratin, whereas vimentin was expressed at similar level as observed in tumor cells grown in macrophage-conditioned medium (Figure 4F). These findings indicated that our IHC results were not affected by the presence of macrophages. These results suggested macrophage-induced EMT in neoplastic cells, however direct contact of these cell types was not required. Thus, control macrophages constitutively secreted EMT activators, and co-culture with neoplastic cells induced further secretion of these proteins.

### B-catenin localization and Wnt proteins expression in canine mammary cancer tissues and xenografts

IHC analyses of β-catenin localization and Wnt-2, Wnt-5a, Dkk-1, ROR-2, p-PKC, and p-JNK expression in CMT-U27 xenograft tumors (which metastasized) indicated the activation of the non-canonical Wnt pathway (Figure S2). The control CMT-U27 cells grown *in vitro* showed β-catenin nuclear localization, elevated ROR-2 expression, and very low JNK phosphorylation *in vitro*, whereas Wnt-2, Wnt-5a, Dkk-1, and phosphorylated PKC were not detected (Figure 2B). Implantation of these cells into nude mice led to decreased nuclear localization of β-catenin and activated Wnt-2, Wnt-5a, Dkk-1, and p-PKC expression (Figure S3). This effect was similar to those observed after culture in macrophage-conditioned medium or co-culture with TAMs. Considering that these xenograft tumors were exposed to significant infiltration by macrophages and produced lung metastases, our hypothesis may also be valid *in vivo*. To investigate whether our hypothesis is relevant *ex vivo*, we analyzed β-catenin localization in 50 high-grade metastatic (n = 25) and non-metastatic (n = 25) canine mammary tumors (Table 3). Nuclear β-catenin was undetectable in metastatic tumors, indicating inhibition of the canonical Wnt pathway (Figure 5A, Table 3). In contrast, 23 of 25 non-metastatic tumors had detectable nuclear β-catenin (Figure 5B, Table 3). Previous reports described a negative relationship between nuclear β-catenin, metastasis, and poor outcomes [35]–[37]. Accordingly, loss of nuclear β-catenin expression in metastatic mammary cancers was significantly correlated (p<0.01) with the number of macrophages (Figure 5C, D, and E; Table 3). Moreover, we observed increased expression of Wnt-2 (p<0.001), Wnt-5a (p<0.001), Dkk-1 (p<0.001), and ROR-2 (p<0.001, Figure 6A, B, C and D; Table 3) in metastatic canine mammary tumors compared with non-metastatic tumors. It indicated non-canonical Wnt pathway activation in metastatic tumors.

**Figure 5:** Analysis of β-catenin localization and macrophage numbers in metastatic and non-metastatic canine mammary cancer tissues. Images of canine mammary metastatic and non-metastatic tumors were obtained using an Olympus BX60 microscope (400×). Tissue sections were treated with specific anti-β-catenin and anti-MAC387 antibodies and stained using an Envision kit (Dako, Denmark). Labeled antigens are indicated by brown precipitates. Cytoplasmic and membrane-bound β-catenin is observed in metastatic tumor cells, whereas nuclear β-catenin is prevalent in non-metastatic tumor cells (indicated as asterix). Macrophage infiltration is much greater in metastatic tumors than in non-metastatic tumors. The colorimetric intensities of 10–20 images of immunohistochemical-stained antigen spots were counted using a computer-assisted image analyzer (Olympus Microimage™ Image Analysis version 4.0 software for Windows, USA) and were expressed as mean pixel integrated optical density (IOD). Statistical analysis was performed using Prism version 5.00 software (GraphPad Software, USA). Analysis of variance and Tukey's post-hoc tests were applied to identify significant differences in optical density between cell lines. Differences were considered significant when *p<0.05 and highly significant when **p≤0.01 or ***p≤0.001. Spearman's coefficient was used to assess correlations.

**Figure 6:** Analysis of Wnt proteins expression in metastatic and non-metastatic canine mammary cancer tissues. Images showing Wnt-2, Wnt-5a, Dkk-1, and ROR-2 expression in metastatic and non-metastatic canine mammary tumors were obtained using an Olympus BX60 microscope (400×). Tissue sections were treated with specific antibodies and stained using an EnVision kit (Dako, Denmark). Labeled antigens are indicated by brown precipitates. Metastatic tumors show significantly higher expression of all examined antigens compared with non-metastatic tumors. Colorimetric intensities of immunohistochemical-stained antigen spots on 10–20 images were counted using a computer-assisted image analyzer (Olympus Microimage™ Image Analysis version 4.0 software for Windows, USA) and were expressed as mean pixel integrated optical density (IOD). Statistical analysis was performed using Prism version 5.00 software (GraphPad Software, USA). Analysis of variance and Tukey's post-hoc tests were used to identify differences in optical density. Differences were considered significant when *p<0.05, and highly significant when **p≤0.01 or ***p≤0.001.

The canonical Wnt signaling pathway has been implicated in the pathogenesis of several tumor types, promoting proliferation and manifesting in both cytoplasmic and nuclear β-catenin accumulation [38], [39]. However, little is known of the roles and mechanisms of non-canonical Wnt pathways in tumorigenesis. It is supposed to increase cell ability to migration. Previous studies showed that Wnt-5a (non-canonical Wnt activator) overexpression is associated with the migration and invasiveness of several cancers, including gastric, pancreatic, and breast cancers [40]–[43]. Both canonical and non-canonical Wnt pathways show competitive inhibition.

It has also been suggested that during tumor progression, the switch between canonical and non-canonical Wnt signaling pathways might lead to metastasis [44]. However, it has not been linked with the presence or activity of macrophages. Taken together, our results indicate that TAMs induce the switch between canonical and non-canonical Wnt pathways, and thereby inhibit proliferation but promote metastasis in canine mammary tumors (Figure 7). Interestingly, similar changes in neoplastic cells were observed after the addition of macrophage-conditioned medium, indicating that macrophages secrete canonical Wnt inhibitors without stimulation by neoplastic cells. We confirmed that control macrophages secrete the same canonical Wnt inhibitors (Dkk-1, Wnt-2, Wnt-5a) as TAMs but at lower level. Nonetheless, co-culture with tumor cells increases this effect due to their direct contact and thus stimulation by neoplastic cells. We showed that constitutively secreted canonical Wnt inhibitors hamper cancer proliferation and development what prove anti-neoplastic activity of macrophages and refute the “corruption” theory. However, as a side effect macrophages activate non-canonical Wnt signaling and promote metastasis. Understanding of metastasis at the molecular level is of a great therapeutic importance. Although the roles of the tumor microenvironment are increasingly evident in cancer metastasis, only anti-angiogenic therapies are currently available to exploit this. There are also some reports available about experimental anti-macrophage treatment [45], [46] for metastatic cancers. However, the present data suggests that the modulation of TAMs activity may offer superior therapeutic efficacy.

**Figure 7:** Canonical and non-canonical Wnt pathways. Scheme of the interactions observed between canonical and non-canonical Wnt pathways.

## Conclusions

This is the first study to show that TAMs mediate a switch between canonical and non-canonical Wnt signaling in canine mammary tumors. Based on the results of our studies we hypothesize that macrophages infiltrating tumor mass secrete canonical Wnt inhibitors in order to hamper cancer proliferation and development but as a side effect they activate non-canonical Wnt signaling and promote metastasis. Thus, although anti-macrophage treatments may undermine the anti-proliferative roles of macrophages, modulation of their activities might offer an efficacious therapeutic strategy. However, more studies in this field are required.

## Supporting Information

Figure S1 Validation of microarray results. Relative expression of two microRNAs: miR-182 (A) and miR-130a (B) in co-cultured and monocultured canine mammary neoplastic cells and macrophages examined using Real-time RT-PCR.
(TIF)

Figure S2 Integrated Optical Density of examined Wnt proteins. The level of examined Wnt proteins was expressed as IOD (Integrated Optical Density) in arbitrary units with the value obtained using the Odyssey Infrared Imaging System (LI-COR Inc., USA). The results are expressed as the mean ±SD. The **ANOVA +** Tukey post-hoc test were applied (Graph Pad v. 5.0), the values differed significantly (p<0.05) were marked as *, whereas values differed highly significant (p<0.01 or p<0.001) were marked as ** or ***, respectively.
(TIF)

Figure S3 Expression of selected Wnt proteins and number of macrophages examinedin CMT-U27 xenograft tumors. Light micrographs of nude mice CMT-U27 xenograft tumors [20] were obtained using an Olympus BX60 microscope (400×); presence of macrophages, β-catenin localization and Wnt-2, Wnt-5a, Dkk-1, ROR-2, p-PKC, and JNK expression in cancer cells. Labeled antigens are indicated by brown precipitates in the cytoplasm and nucleus.
(TIF)

Table S1 MicroRNAs significantly down and up (bold) regulated in tumor cells or macrophages grown as co-culture compared with monoculture. Unpaired t-tests with a Benjamin–Hochberg false discovery rate (FDR) of <5% correction were applied, with a p value cut-off of <0.01, fold change>1.2.
(DOC)

Table S2 Seven highly significant cellular pathways in which are involved miRNA-targeted genes in tumor cells and macrophages grown as co-culture (PANTHER analysis). The analysis revealed that Wnt signaling predominated in both co-cultured cell types.
(DOC)
